The article "Plant-growth-promoting Bacillus and Paenibacillus species improve the nutritional status of Triticum aestivum L" was retracted in 2023. Reasons: original data or images not available; a conflict of interest; concerns about the peer review; concerns about the citations.

# Plant-growth-promoting *Bacillus* and *Paenibacillus* species improve the nutritional status of *Triticum aestivum* L.

**DOI:** 10.1371/journal.pone.0241130

**Published:** 2020-12-01

**Authors:** Azhar Hussain, Maqshoof Ahmad, Muhammad Nafees, Zafar Iqbal, Muhammad Luqman, Moazzam Jamil, Ambreen Maqsood, Freddy Mora-Poblete, Sunny Ahmar, Jen-Tsung Chen, Mohammed Nasser Alyemeni, Parvaiz Ahmad

**Affiliations:** 1 Department of Soil Science, The Islamia University of Bahawalpur, Bahawalpur, Pakistan; 2 Department of Horticultural Sciences, The Islamia University of Bahawalpur, Bahawalpur, Pakistan; 3 Department of Plant Pathology, The Islamia University of Bahawalpur, Bahawalpur, Pakistan; 4 Institute of Biological Sciences, University of Talca, Talca, Chile; 5 College of Plant Science and Technology, Huazhong Agricultural University, Wuhan, China; 6 Department of Life Sciences, National University of Kaohsiung, Kaohsiung, Taiwan; 7 Botany and Microbiology Department, College of Science, King Saud University, Riyadh, Saudi Arabia; 8 Department of Botany, S.P. College, Srinagar, Jammu and Kashmir, India; Universite d’Orleans, FRANCE

## Abstract

Wheat is one of the best-domesticated cereal crops and one of the vital sources of nutrition for humans. An investigation was undertaken to reveal the potential of novel bio-inoculants enriching micronutrients in shoot and grains of wheat crop to eliminate the hazards of malnutrition. Sole as well as consortia inoculation of bio-inoculants significantly enhanced mineral nutrients including zinc (Zn) and iron (Fe) concentrations in shoot and grains of wheat. Various treatments of bio-inoculants increase Zn and Fe content up to 1–15% and 3–13%, respectively. Sole inoculation of *Bacillus aryabhattai* (S10) impressively improves the nutritious of wheat. However, the maximum increase in minerals contents of wheat was recorded by consortia inoculation of *Paenibacillus polymyxa* ZM27, *Bacillus subtilis* ZM63 and *Bacillus aryabhattai* S10. This treatment also showed a maximum bacterial population (18 × 10^4^ cfu mL^-1^) in the rhizosphere. The consortium application of these strains showed up to a 17% increase in yield. It is evident from the results that the consortium application was more effective than sole and co-inoculation. A healthy positive correlation was found between growth, yield, and the accessibility of micronutrients to wheat crops at the harvesting stage. The present investigations revealed the significance of novel bacterial strains in improving the nutritional status of wheat crops. These strains could be used as bio-inoculants for the biofortification of wheat to combat hidden hunger in developing countries.

## 1. Introduction

Wheat (*Triticum aestivum* L.) is the staple food for more than 35% population of the world [1]. Wheat is the only diet in many nutrient-deficient regions worldwide [2]. Global food production has improved by many folds as associated with the past, but the static pace of agriculture development is not satisfactory for the rapidly increasing population [3]. Sustainable wheat production requires suitable amounts of chemical fertilizers. However, it is usually practiced in excessive amounts causing a negative impact on the environmental and high cost associated with environmental management. Moreover, in recent era concerning human health scientists tried to find a resurgence of sustainable and environmentally friendly agriculture [4].

In developing countries, malnutrition is a major threat to human health [5]. Children and women are mostly affected by malnutrition [6]. About 40% of the women and children population in the world has been reported with a deficiency of Fe, caused anemia and weak immune system [5]. It is estimated that about 75% of the world’s population suffers from an inadequate supply of micronutrients in diet including Zn, Cu, and Fe [6–8]. Consequently, inadequate supply of Zn and Cu caused respiratory and digestive disorders, fatigue, high blood pressure, and immunity failure [9]. This situation demands that the appropriate measure should be taken to combat malnutrition and avoid human health losses. Micronutrient deficiencies in diet can be cured either by pharmacological supplementation or through agriculture-based micronutrient biofortification.

Biofortification is a sustainable food-based technique to combat micronutrient deficiencies in humans [10]. Biofortification by following agronomic practices along with molecular breeding techniques are being advocated to tackle malnutrition worldwide [11]. Injudicious use of chemical fertilizers to meet world food demands has given rise to diminished accumulation of Zn and Fe in cereal grains. As Zn and Fe both are the significant micronutrients for a balanced human diet [12]. Being a staple food for a large proportion of the world’s population, the deficiency of these nutrients in wheat has serious consequences. Therefore, an integrated approach associated with increased micronutrient concentration would be of immense importance to cure malnutrition. Agriculture based biofortification is mostly achieved by direct application of fertilizers to crops. But this approach is not suitable for developing countries because of the high associated cost and long-term application of nutrient fertilizers causing potential risks to the environment. Contrarily plant growth-promoting bacteria are known to cause increased micronutrient concentrations in plants including Fe and Zn [6,13]. These microbes when applied to the soil ultimately enhance plant growth by improving nutrients solubility, acquisition, and availability to crops [4,14]. The use of PGPR is steadily increasing in agriculture, as it offers an attractive way to reduce the use of chemical fertilizers, pesticides and other agrochemicals. The application of PGPR in the wheat crop has the potential to reduce the use of chemical fertilizer up to 20–50% without compromising the quality of the produce. This ultimately reduces the cost of production [15].

In earlier investigations, we separated and depicted numerous strains from genera *Paenibacillus* and *Bacillus*, in the examination facility. These novel inoculants have been documented as *Bacillus aryabhattai* strain ZM31, *Paenibacillus polymyxa* strain ZM27, *Bacillus aryabhattai* strain S10, and *Bacillus subtilis* strain ZM63 [6] and have been distributed to Gene bank through accession numbers KX788860, KX788859, KX788862, and KX788861, respectively. These novel inoculants have Zn solubilizing capacity along with at least one of the special characters, such as the production of exopolysaccharides, production of indole acetic acid, solubilizing of phosphate, siderophores production, production of ACC- deaminase, catalase activity, and so on. Biofortification of wheat crop by utilizing these potential novel strains can be done to reduce malnutrition in the world. Current investigations energies for a comprehensive assessment of these strains for sustainable production of quality wheat in South Punjab.

## 2. Results

### 2.1. Pot trials

Novel bio-inoculants were tested for their impact on growth parameters of the wheat crop in a pot trial. For this purpose, two pot trials were conducted in the wirehouse of the Department of Soil Science, The Islamia University of Bahawalpur. After 50 days of sowing, growth parameters were recorded, and micronutrient contents were analyzed in the shoot. Findings are present as follows.

#### 2.1.1. Impacts of novel bio inoculants on wheat growth parameters

Novel bio-inoculants had a positive impact on the growth of wheat. Sole inoculation of ZM27 and ZM31 has a nonsignificant influence on growth attributes over control while all other applied treatments significantly improve growth. The consortium application of three strains (ZM27+ZM63+S10) showed maximum plant height followed by the co-inoculation of ZM27+S10. These treatments showed a 53% and 45% increase in plant height, respectively (Fig 1).

**Fig 1:** Effects of novel bio-inoculants on plant height of wheat in a pot trial. Data are present as a mean of three replicates. Bars sharing same letter(s) are statistically similar (*p≤0*.*05*). T_1_; Control, T_2_; ZM27, T_3_; ZM31, T_4_; ZM63, T_5_; S10, T_6_; ZM27 + ZM31, T_7_; ZM27 + ZM63, T_8_; ZM27 + S10, T_9_; ZM31 + ZM63, T_10_; ZM31 + S10, T_11_; ZM63 + S10, T_12_; ZM27 + ZM31 + ZM63, T_13_; ZM27 + ZM31 + S10, T_14_; ZM27 + ZM63 + S10, T_15_; ZM31 + ZM63 + S10, T_16_; ZM27 + ZM31 + ZM63 + S10.

Sole application of S10 showed a significant impact on improving shoot dry biomass which was 27% more than control. While the maximum 47% increase in shoot dry biomass was found by the consortium application of ZE27+ZM63+S10. Co-inoculation of ZM27+S10 was the next treatment which showed a 40% increase in shoot dry biomass (Fig 2). Minimum root dry biomass was observed 1.23 g plant^-1^ in un-inoculated control, whereas maximum root dry biomass (2.43 g plant^-1^) was found by the consortium application of ZE27+ZM63+S10 (Fig 3).

**Fig 2:** Effects of novel bio-inoculants on shoot dry biomass of wheat in a pot trial. Data are present as a mean of three replicates. Bars sharing same letter(s) are statistically similar (*p≤0*.*05*). T_1_; Control, T_2_; ZM27, T_3_; ZM31, T_4_; ZM63, T_5_; S10, T_6_; ZM27 + ZM31, T_7_; ZM27 + ZM63, T_8_; ZM27 + S10, T_9_; ZM31 + ZM63, T_10_; ZM31 + S10, T_11_; ZM63 + S10, T_12_; ZM27 + ZM31 + ZM63, T_13_; ZM27 + ZM31 + S10, T_14_; ZM27 + ZM63 + S10, T_15_; ZM31 + ZM63 + S10, T_16_; ZM27 + ZM31 + ZM63 + S10.

**Fig 3:** Effects of novel bioinoculants on root dry biomass of wheat in a pot trial. Data are present as a mean of three replicates. Bars sharing same letter(s) are statistically similar (*p≤0*.*05*). T_1_; Control, T_2_; ZM27, T_3_; ZM31, T_4_; ZM63, T_5_; S10, T_6_; ZM27 + ZM31, T_7_; ZM27 + ZM63, T_8_; ZM27 + S10, T_9_; ZM31 + ZM63, T_10_; ZM31 + S10, T_11_; ZM63 + S10, T_12_; ZM27 + ZM31 + ZM63, T_13_; ZM27 + ZM31 + S10, T_14_; ZM27 + ZM63 + S10, T_15_; ZM31 + ZM63 + S10, T_16_; ZM27 + ZM31 + ZM63 + S10.

#### 2.1.2. Accumulation of Fe and Zn in the shoot of wheat

Sole as well as consortium application of novel bio-inoculant of plant growth-promoting rhizobacteria improve iron and zinc contents in the shoot of wheat. In both trials, inoculated treatments expressed excellent results regarding the improvement of Fe and Zn contents as compared to un-inoculated control (Table 1). A maximum 15% increase in Fe content was observed by the co-inoculation of ZM27+S10. While the maximum 12% increase in Zn content was recorded by the consortium application of ZM27+ZM63+S10. The co-inoculation of ZM27+S10 and consortium application of ZM27+ZM63+S10 exhibited 10% and 14% in Zn and Fe content, respectively.

**Table 1:** Effects of novel bio-inoculants on bacterial population in rhizosphere and iron & zinc content in the shoot of wheat in a pot trial.

Treatments	Bacterial population (cfu × 10^4^)		Fe content (mg kg^-1^)		Zn content (mg kg^-1^)	
	Trial I	Trial II	Trial I	Trial II	Trial I	Trial II
Control	38.7 e	40.3 f	10.02 i	10.21 e	14.10 f	13.64 d
ZM27	39.3 e	41.7 ef	10.34 hi	10.46 de	14.23 ef	13.72 d
ZM31	39.3 e	42.3 ef	10.59 f-h	10.54 c-e	14.21 f	13.80 d
ZM63	40.3 de	42.3 ef	10.69 e-h	10.55 c-e	14.45 d-f	13.84 d
S10	41.0 de	41.0 ef	10.53 gh	10.65 b-e	14.32 ef	14.00 cd
ZM27+ZM31	41.0 de	42.3 ef	10.55 gh	10.71 b-d	14.68 de	14.15 b-d
ZM27+ZM63	41.7 de	44.0 d-f	10.55 gh	10.68 b-d	14.31 ef	14.09 b-d
ZM27+S10	45.0 b-d	49.7 ab	11.51 a	11.05 ab	15.53 ab	14.71 a
ZM31+ZM63	42.7 c-e	45.0 c-e	10.79 d-h	10.75 a-d	15.43 ab	14.39 a-c
ZM31+S10	43.7 c-e	45.0 c-e	10.72 e-h	10.80 a-d	14.85 cd	14.53 ab
ZM63+S10	43.3 c-e	47.0 b-d	11.02 b-f	10.67 b-e	14.86 cd	14.50 a-c
ZM27+ZM31+ZM63	45.0 b-d	49.3 a-c	10.94 c-g	10.72 b-d	15.43 ab	14.52 ab
ZM27+ZM31+S10	44.0 c-e	50.7ab	11.09 a-e	10.74 b-d	15.24 bc	14.59 ab
ZM27+ZM63+S10	48.0 a-c	53.7 a	11.42 ab	11.22 a	15.79 a	14.86 a
ZM31+ZM63+S10	50.7 a	49.7 ab	11.23 a-d	10.96 a-c	15.46 ab	14.68 a
ZM27+ZM31+ZM63+S10	49.7 ab	48.7 bc	11.29 a-c	10.80 a-d	15.50 ab	14.76 a
LSD (p≤0.05)	5.3463	4.3937	0.4697	0.4698	0.4651	0.5198

Data are present as mean of three replicates. Means followed by same letter(s) within a column are statistically similar (*p≤0*.*05*). cfu; colony forming unit.

#### 2.1.3. Application of novel bio inoculants improve bacterial population

The viability of the individual and combined application of bacterial strains on the bacterial population in the rhizosphere of wheat depicted in Table 1). In both pot trials, the bacterial population increased essentially by inoculation as compared to un-inoculated control. Co-inoculation with ZM27+ S10 showed a 23% increment over un-inoculated control in the trial II while a 16% increase was observed in the trial I. Consortia application of ZM27+ZM31+S10 revealed a maximum 33% and 26% increase in the bacterial population in the trial I and II, respectively.

### 2.2. Field trial

To confirm the results of pot trials, these strains were further evaluated under field conditions for growth, yield, and biofortification of wheat grain. For this purpose, four field trials were conducted in the research area of the Department of Soil Science, The Islamia University of Bahawalpur. The results of field trials are described below as;

#### 2.2.1. Plant height and shoot dry biomass improved by novel bio inoculants

Sole as well as the combined application of plant growth-promoting rhizobacteria (PGPR) strains improved plant height as compared to un-inoculated control (Table 2). Consortia application of bacterial strains showed more promising results than sole and co-inoculation. Maximum 23%, 17%, 22%, and 19% in plant height was observed due to consortium application of ZM27+ZM63+S10 in field trials I to IV, respectively. Among co-inoculation, ZM27+S10 showed better results than all other co-inoculated treatments where a 19% increase in plant height was observed in the trial I while in all the other three trials 16% increase was observed. Among sole inoculation, S10 has maximum influenced on plant height. All applied treatments of novel bio inoculants significantly enhanced shoot dry biomass in all field trials (Table 2). Sole inoculation gave up to 14% increase in shoot dry biomass while with co-inoculation up to 20% increase in shoot dry biomass was recorded as compared to un-inoculated control. A maximum of 29% increase in shoot dry biomass was observed due to the consortia application of ZM27+ZM63+S10. A consortium application where all strain was applied collectively (ZM27+ZM31+ZM63+S10) was the next treatment to improve shoot dry biomass which showed up to 26% increase in shoot dry biomass.

**Table 2:** Effects of novel bio-inoculants on plant height and shoot dry biomass of wheat in a field trial.

Treatments	Plant height (cm)				Shoot dry biomass (g plant^-1^)			
	Trial I	Trial II	Trial III	Trial IV	Trial I	Trial II	Trial III	Trial IV
Control	70.0 g	69.0 g	72.0 e	71.3 e	4.47 d	5.53 c	5.62 d	5.08 e
ZM27	73.7 fg	72.0 e-g	75.0 de	77.0 d	4.90 b-d	5.72 bc	6.00 b-d	5.19 de
ZM31	75.0 ef	71.7 fg	74.3 de	76.0 de	4.85 b-d	5.85 a-c	5.82 cd	5.57 b-e
ZM63	76.0 d-f	73.3 d-g	76.7 cd	77.7 cd	4.68 cd	5.80 bc	5.97 b-d	5.50 b-e
S10	78.7 c-e	75.3 c-f	77.7 cd	76.7 de	5.08 a-d	5.84 a-c	6.05 a-d	5.76 a-e
ZM27+ZM31	77.0 d-f	75.3 c-f	78.0 cd	79.3 b-d	5.03 a-d	5.69 bc	6.09 a-d	5.65 b-e
ZM27+ZM63	77.3 d-f	75.0 c-f	80.7 bc	79.7 b-d	5.20 a-d	6.00 a-c	6.31 a-d	5.37 c-e
ZM27+S10	83.0 ab	80.3 ab	83.7 ab	83.3 ab	5.22 a-d	6.18 a-c	6.58 a-d	6.02 a-c
ZM31+ZM63	78.7 c-e	77.7 a-d	80.0 bc	80.3 a-d	5.08 a-d	5.92 a-c	6.32 a-d	5.83 a-e
ZM31+S10	76.3 d-f	76.3 b-e	80.3 bc	81.0 a-d	5.15 a-d	6.15 a-c	6.49 a-d	5.97 a-c
ZM63+S10	77.7 de	75.7 c-f	81.0 bc	81.3 a-d	5.35 a-c	5.98 a-c	6.33 a-d	5.81 a-e
ZM27+ZM31+ZM63	79.3 b-d	78.0 a-c	83.7 ab	83.7 ab	5.35 a-c	6.39 a-c	6.47 a-d	5.91 a-d
ZM27+ZM31+S10	78.0 de	76.0 b-f	81.0 bc	81.3 a-d	5.52 ab	6.51 a-c	6.75 a-c	6.14 ab
ZM27+ZM63+S10	86.3 a	81.0 a	88.0 a	85.3 a	5.77 a	6.92 a	7.03 a	6.48 a
ZM31+ZM63+S10	82.3 bc	77.3 a-d	83.7 ab	81.3 a-d	5.41 a-c	6.69 ab	6.81 a-c	6.27 ab
ZM27+ZM31+ZM63+S10	79.7 b-d	77.0 a-d	81.0 bc	82.7 a-c	5.58 ab	6.42 a-c	6.90 ab	6.42 a
LSD (p≤0.05)	3.8045	4.3789	4.5671	5.4803	0.7839	1.0860	1.0016	0.7688

Data are present as mean of three replicates. Means followed by same letter(s) within a column are statistically similar (*p≤0*.*05*).

#### 2.2.2. Novel bio inoculants significantly improve the yield of wheat

The results revealed that the application of novel bio-inoculants separately and in combination has a positive influence on yield attributes of wheat crop. All treatment of sole as well as the combined application of PGPR were significantly increased 1000 grain weight of wheat in all field trials except ZM27 in field trial II where it showed non-significant results (Table 3). The co-inoculation resulted in a significantly higher increase in 1000 grain weight as compared to sole inoculation. Furthermore, the combined use of ZM27+ZM63+S10 showed the maximum increase (up to 11%) in 1000 grain weight when compared with un-inoculated control. The maximum increase in grain yield was observed due to the consortium application of ZM27+ZM63+S10, where up to a 17% increase was observed as compared to un-inoculated control (Table 4). Among co-inoculation combinations, ZM27+S10 showed up to a 15% increase in grain yield. Furthermore, the sole application of PGPR also significantly increased the grain yield as compared to un-inoculated control. Sole as well as the combined application of PGPR significantly enhanced straw yield in all field trials, but sole inoculation of ZM27 in field trial III showed non-significant results as compared to un-inoculated control (Table 4). Among sole inoculation, S10 showed better results as compared to other sole inoculated treatments. However, the maximum increase in straw yield up to16% was observed due to the consortium application of ZM27+ZM63+S10.

**Table 3:** Effects of novel bio-inoculants on bacterial population in rhizosphere and 1000-grain weight of wheat in a field trial.

Treatments	Bacterial population (cfu × 10^4^)				1000-grain weight (g)			
	Trial I	Trial II	Trial III	Trial IV	Trial I	Trial II	Trial III	Trial IV
Control	25.5 e	24.0 c	23.3 c	23.3 c	39.8 i	39.5 g	40.1 h	39.0 f
ZM27	26.5 de	26.3 bc	25.3 bc	25.0 bc	40.0 hi	40.1 fg	40.2 h	40.0 ef
ZM31	27.2 b-e	26.3 bc	24.7 bc	26.0 a-c	40.7 g-i	40.1 fg	40.7 gh	39.6 ef
ZM63	26.8 c-e	26.7 bc	25.3 bc	25.7 a-c	40.9 f-h	40.5 e-g	40.7 f-h	40.5 de
S10	28.0 b-e	27.0 a-c	25.7 bc	26.3 a-c	41.2 e-g	40.3 e-g	40.8 f-h	41.2 cd
ZM27+ZM31	27.8 b-e	27.3 a-c	26.3 a-c	25.7 a-c	42.1 b-e	40.8 b-f	42.0 de	41.1 cd
ZM27+ZM63	28.8 a-e	27.0 a-c	26.7 a-c	25.7 a-c	41.5 d-g	41.5 c-e	41.6 e-g	40.4 de
ZM27+S10	30.3 ab	29.3 ab	27.7 ab	28.3 ab	42.4 b-d	42.0 b-d	42.2 c-e	42.1 a-c
ZM31+ZM63	29.2 a-d	27.3 a-c	26.3 a-c	26.7 a-c	42.3 b-d	41.9 b-d	41.3 e-g	42.0 a-c
ZM31+S10	28.7 a-e	27.3 a-c	26.7 a-c	26.3 a-c	42.3 b-d	41.8 b-d	41.8 d-f	41.7 bc
ZM63+S10	30.5 ab	28.0 a-c	27.0 a-c	27.0 a-c	41.8 c-f	42.0 b-d	42.3 c-e	41.8 a-c
ZM27+ZM31+ZM63	30.0 a-c	27.7 a-c	27.3 ab	27.3 ab	42.7 a-c	42.6 bc	43.1 a-c	42.0 a-c
ZM27+ZM31+S10	29.7 a-d	28.3 ab	27.3 ab	26.3 a-c	42.5 b-d	42.0 b-d	42.8 b-d	42.2 a-c
ZM27+ZM63+S10	31.7 a	31.0 a	29.7 a	29.3 a	43.6 a	44.0 a	44.0 a	42.9 a
ZM31+ZM63+S10	30.3 ab	29.0 ab	28.0 ab	28.0 ab	42.7 a-c	43.0 ab	43.5 ab	42.5 ab
ZM27+ZM31+ZM63+S10	28.7 a-e	29.3 ab	27.7 ab	27.3 ab	43.0 ab	43.1 ab	43.1 a-c	41.9 a-c
LSD (*p≤0*.*05*)	3.3564	4.0963	3.9072	3.9426	1.0371	1.2415	1.0713	1.1227

Data are present as mean of three replicates. Means followed by same letter(s) within a column are statistically similar (*p≤0*.*05*). cfu; colony forming unit.

**Table 4:** Effects of novel bio-inoculants on grain and straw yield of wheat in a field trial.

Treatments	Grain yield (tons ha^-1^)				Straw yield (tons ha^-1^)			
	Trial I	Trial II	Trial III	Trial IV	Trial I	Trial II	Trial III	Trial IV
Control	4.68 i	4.70 j	4.82 h	4.77 h	5.09 h	5.39 i	5.44 f	5.36 i
ZM27	4.84 gh	4.80 ij	4.98 g	5.02 g	5.18 gh	5.62 h	5.46 f	5.58 gh
ZM31	4.75 hi	4.81 h-j	5.04 fg	5.00 g	5.26 fg	5.63 h	5.58 d-f	5.52 h
ZM63	4.80 g-i	4.82 hi	5.01 g	5.03 fg	5.17 gh	5.64 h	5.53 ef	5.62 f-g
S10	4.89 fg	4.92 gh	5.10 e-g	5.19 de	5.27 fg	5.74 gh	5.68 c-e	5.71 f
ZM27+ZM31	4.91 fg	4.97 fg	5.15 ef	5.14 e	5.32 f	5.79 fg	5.63 de	5.73 f
ZM27+ZM63	4.84 gh	4.90 g-i	5.08 fg	5.13 ef	5.35 ef	5.72 gh	5.70 cd	5.65 fg
ZM27+S10	5.16 bc	5.22 bc	5.40 bc	5.47 b	5.57 bc	6.04 b-d	5.95 b	6.06 bc
ZM31+ZM63	5.03 de	5.09 de	5.27 d	5.26 cd	5.44 de	5.91 d-f	5.82 bc	5.91 de
ZM31+S10	4.97 ef	5.03 ef	5.22 de	5.30 c	5.45 de	5.85 e-g	5.83 bc	5.89 e
ZM63+S10	5.21 b	5.17 b-d	5.45 b	5.42 b	5.52 b-d	5.99 b-e	5.84 bc	6.01 b-d
ZM27+ZM31+ZM63	5.05 c-e	5.11 c-e	5.30 cd	5.26 cd	5.46 cd	5.93 c-e	5.88 b	5.91 de
ZM27+ZM31+S10	5.20 b	5.26 b	5.45 b	5.49 b	5.61 b	6.08 b	5.93 b	6.11 b
ZM27+ZM63+S10	5.35 a	5.41 a	5.60 a	5.60 a	5.76 a	6.23 a	6.11 a	6.23 a
ZM31+ZM63+S10	5.12 b-d	5.23 b	5.41 bc	5.42 b	5.58 bc	6.05 b-d	5.96 ab	5.99 b-e
ZM27+ZM31+ZM63+S10	5.18 b	5.24 b	5.49 ab	5.46 b	5.59 b	6.06 bc	5.94 b	6.05 bc
LSD (*p≤0*.*05*)	0.1193	0.1129	0.1232	0.1010	0.1154	0.1368	0.1576	0.1150

Data are present as mean of three replicates. Means followed by same letter(s) within a column are statistically similar (*p≤0*.*05*).

#### 2.2.3. Biofortification of wheat grain through novel bio inoculants

The inoculation with novel PGPR strains significantly improved the Fe and Zn concentration in wheat grains under field conditions at all experimental sites when compared with uninoculated control (Table 5). The sole application of S10 resulted in up to a 5% increase in iron concentration. The combined application of ZM27+ZM63+S10 increased the iron concentration in wheat grains up to 13%. All treatment showed a significant increase in zinc concentration in wheat grains in all field trials except ZM27 which showed no-significant results in field trial I & IV as compared to un-inoculated control (Table 6). Individual application of S10 resulted in up to a 7% increase in zinc concentration in grains of wheat. The co-inoculation of ZM27+S10 and ZM63+S10 showed better results as compared to the sole application that resulted in up to 10% and 9% increase in zinc concentration, respectively. The combined application of PGPR strains showed significantly better results than individual applications. A maximum increase in zinc concentration in wheat grains up to 15% was observed due to the consortium application of ZM27+ZM63+S10. The overall results showed that the combined use of bacterial strains was more effective than the sole application of these strains.

**Table 5:** Effects of novel bio-inoculants on iron and zinc content in grains of wheat in a field trial.

Treatments	Fe content in grain (mg kg^-1^)				Zn content in grain (mg kg^-1^)			
	Trial I	Trial II	Trial III	Trial IV	Trial I	Trial II	Trial III	Trial IV
Control	11.2 f	10.4 j	8.27 g	8.88 j	6.99 j	7.50 j	8.89 k	8.77 k
ZM27	11.5 d-f	10.5 ij	8.73 d-f	8.96 ij	7.06 j	7.60 i	9.12 j	8.82 k
ZM31	11.8 b-f	10.5 i	8.55 e-g	9.16 fg	7.23 i	7.66 i	9.26 i	8.91 j
ZM63	11.3 ef	10.4 ij	8.61 ef	9.08 gh	7.31 h	7.79 h	9.29 i	9.11 h
S10	11.6 c-f	10.5 hi	8.67 ef	9.03 hi	7.51 f	7.75 h	9.52 gh	9.02 i
ZM27+ZM31	11.8 b-f	10.7 gh	8.46 fg	9.14 g	7.46 f	7.87 g	9.59 fg	9.23 g
ZM27+ZM63	11.6 c-f	10.7 fg	8.97 b-d	9.25 ef	7.39 g	8.04 f	9.45 h	9.33 f
ZM27+S10	12.1 a-d	10.9 de	9.06 bc	9.57 c	7.83 c	8.28 d	9.79 c-e	9.52 c
ZM31+ZM63	12.0 a-e	10.8 ef	8.98 b-d	9.35 de	7.64 e	8.18 e	9.74 e	9.40 e
ZM31+S10	11.7 b-f	10.6 hi	8.78 c-e	9.44 d	7.62 e	8.15 e	9.66 f	9.43 de
ZM63+S10	12.1 a-d	11.1 c	9.06 bc	9.58 c	7.73 d	8.20 e	9.75 de	9.60 b
ZM27+ZM31+ZM63	12.3 a-c	11.1 bc	8.98 b-d	9.88 a	7.75 d	8.36 c	9.94 b	9.53 c
ZM27+ZM31+S10	12.2 a-d	11.0 cd	9.19 ab	9.63 c	7.88 bc	8.38 c	9.86 c	9.47 cd
ZM27+ZM63+S10	12.7 a	11.3 a	9.36 a	9.98 a	8.06 a	8.56 a	10.05 a	9.72 a
ZM31+ZM63+S10	12.5 ab	11.2 ab	9.14 ab	9.77 b	7.93 b	8.47 b	9.96 b	9.63 b
ZM27+ZM31+ZM63+S10	12.0 a-e	11.0 cd	8.99 b-d	9.61 c	7.82 c	8.36 c	9.82 cd	9.49 cd
LSD (*p≤0*.*05*)	0.8038	0.1152	0.2912	0.1007	0.0703	0.0721	0.0731	0.0621

Data are present as mean of three replicates. Means followed by same letter(s) within a column are statistically similar (*p≤0*.*05*).

**Table 6:** Physico-chemical characteristics of the soil prior to sowing.

Parameter	Unit	Pot trials	Field trial I	Field trial II	Field trial III	Field trial IV
**EC**_**e**_	dS m^-1^	1.9	2.1	1.9	1.9	1.6
**pH**	---	7.8	8.1	7.9	7.8	7.7
**Organic matter**	%	0.43	0.41	0.39	0.44	0.48
**N**	%	0.058	0.048	0.043	0.051	0.056
**P**	mg kg^-1^	4.0	3.7	4.2	4.1	5.0
**K**	mg kg^-1^	81	63	71	73	65
**Saturation percentage**	%	35	35	36	36	34
**Textural class**	---	Sandy loam	Sandy loam	Sandy loam	Sandy loam	Sandy loam

#### 2.2.4. Application of novel bio inoculants improve bacterial population

Results regarding bacterial population in wheat rhizosphere under field conditions are presented in Table 3. Sole as well as the combined application of PGPR strains significantly increase the bacterial population in the rhizosphere of wheat at all experimental sites. Among sole inoculation, S10 showed up to a 10% increase in the bacterial population. However, the combined application of PGPR showed better results than sole inoculation. The consortium application of ZM27+ZM63+S10 showed a maximum increase of up to 29% in the bacterial population as compared to the uninoculated control.

## 3. Discussion

In the present study, novel bio-inoculants of plant growth-promoting rhizobacterial strains were evaluated as sole as well as consortia application for their biofortification potential in wheat crops. These bacterial strains can sustain in soil and fix atmospheric nitrogen into the soil. Ultimately increased nitrogen contents in soil by the novel PGPB increase the soil fertility status. The application of bio-inoculants on the crop is an auspicious way of accomplishing sustainability and productivity in agriculture [16–18].

Unfair usage of chemical fertilizers and reduction in the application of organic amendments in crops has steered to the deficiency of micro and macronutrients and diminishing of the chemical, physical and biological characteristics of soil [19–21]. Inoculation of wheat seed with selected bacterial strains, *Paenibacillus polymyxa* (ZM27), *Bacillus subtilis* (ZM63), *Bacillus aryabhattai* (ZM31), and *Paenibacillus polymyxa* (S10), was found excellent to elevate plant development such as increasing minerals in grains and shoot of wheat crop.

In current findings, improved plant growth statuses due to the application of novel bio-inoculants in individuals as well as in consortium were noted. These consequences are sustained by various investigations. The biofertilizer utilization has already been proved to increase in plant development in Zahir *et al*. [22] investigations. Like our outcomes, Zafar-ul-Hye *et al*. [23] additionally defended our findings who concluded that, deployment of biofertilizer along with natural manure extraordinarily reformed the vegetative improvement of plants. The improved plant characteristics are may be due to the potential of novel bio-inoculants of plant growth-promoting rhizobacteria to solubilize the insoluble minerals, to fix atmospheric nitrogen and due to other plant growth and nutritional enrichment qualities which have been proven from our previous study [6]. Nutrient approachability that enhances plant developmental processes has been revealed Ahmad *et al*. [24] by proper consumption of biofertilizer. Current findings upheld by Zafar-ul-Hye *et al*. [23] and Zahir *et al*. [22], who concluded that the exploitation of biofertilizer, improves plant vegetative growth.

Four novel bio-inoculant bacterial strains were additionally tested to assess their PGP and fortification investigation in wheat crops. The impact of bacterial strains on plant height was evidently increased in pots and field experiments. Among individual application of four strains, *Paenibacillus polymyxa* (S10) proved high increment in plant height as well as shoot dry biomass over to un-inoculated control. While among the consortia application of novel inoculants of PGPR, *Bacillus aryabhattai* (S10) + *Paenibacillus polymyxa* (ZM27) + *Bacillus subtilis* (ZM63) was found to enhance the plant growth parameters. The bacterial population in the rhizosphere was remarkably found improving rhizospheric properties by the utilization of novel inoculants. In our investigations, novel inoculants application sole, as well as consortia form, showed their potential for improving Zn and Fe contents in wheat. These results are supported by several studies. Similar to our study, Zahir *et al*. [22] reported the increase in growth attributes due to the application of biofertilizers. Zafar-ul-Hye *et al*. [23] also supported our finding who reported that the application of organic fertilizer along with biofertilizer significantly improved the vegetative growth of the plant. The application of biofertilizer increases nutrient availability that leads to improve growth [24]. The enhancement in plant height, shoot fresh biomass and shoot dry biomass of maize and wheat in response to inoculation with PGPR has been previously reported by Khalid *et al*. [25].

Proper handling of bio-inoculants was noted for improving the available micronutrient content in grains and plant shoots at the harvesting stage. Sole application of *Paenibacillus polymyxa* (S10) was remarkably noted for improving Zn and Fe contents in grains and shoot of wheat which has been comprehensively presented in results. While consortia application of *Paenibacillus polymyxa* (S10) with *Paenibacillus polymyxa* (ZM27), *Bacillus subtilis* (ZM63) gave excellent results for enriching Zn and Fe contents as compared to un-inoculated control. These findings are supported by different authors who reported the increase in mineral contents in grains after the application of bio inoculant. The combined application of biofertilizer with biogas slurry results in the improvement of nutrient availability [26–28] reported that the application of organic fertilizers resulted in improved soil organic matter and physical properties and nutrient availability which enhance plant growth. The present finding was supported by the work of Zahir *et al*. [22] and Zafar-ul-Hye *et al*. [23], who reported that application of biofertilizer, improved vegetative growth. Our findings are supported by Mumtaz et al., [5] who reported the biofortification of Fe and Zn in maize grain by the application of *bacillus* and *Paenibacillus*. Previous experiments confirm our innovations as Hussain et al., [14] and Mumtaz et al., [9] that the novel inoculation stretched the microbial community in the rhizosphere that ultimately increases the availability of micronutrients to crop plants. Thus; resulted in the enrichment of plant shoot and grains with minerals including Fe and Zn.

## 4. Materials and methods

### 4.1. Selection and preparation of bacterial strains

Pre-isolated bacterial strains *Paenibacillus polymyxa* ZM27, *Bacillus aryabhattai* ZM31, *Bacillus subtilis* ZM63 and *Bacillus aryabhattai* S10 [9] were used as single and their all possible combinations to evaluate their potential for the fortification of wheat grains. Luria-Bertani broth culture (100mL) of each bacterial strain was prepared in a 250mL conical flask and incubate at 30 ± 1°C in a rotary shaker [29]. Wheat seeds were inoculated with 48 hrs old bacterial culture of respective strain. For co-inoculation and consortia inoculation strains were used in a 1:1 ratio.

### 4.2. Pot trials

Two (2) pot experiments were conducted in the wirehouse of the Department of Soil Science, The Islamia University of Bahawalpur. This area is recognized as arid-dry to semi-arid-dry. Pots were filled with 12 kg of soil. Before pot filling, soil samples were collected and analyzed for physicochemical characteristics (Table 6). Pots were arranged in a completely randomized design (CRD) for sixteen (16) treatments with three replicates Proposed amount of P (90 kg ha^-1^) and K (60 kg ha^-1^) each whereas 1/3 amount of the prescribed dose (120 kg ha^-1^) of N was applied as basal dose in the form of diammonium phosphate, sulfate of potash, and urea, respectively. While the remaining dose of nitrogen was given in 2 splits. After 50 days, growth parameters were measures and plants were harvested for micronutrient (Fe and Zn) analyses in the shoot [30]. For this purpose, 1 g dry sample was taken in 100 mL digestion tubes followed by 10 mL di-acid mixture (HNO_3_-HCl; 2:1 ratio) and keep it overnight. Next day, heat the tubes in block digester for one hour at 150°C. Then gradually raise temperature up to 235°C and heat for 30 minutes at a constant temperature. After cooling, digested samples were diluted with distilled water. Absorbance reading were measured by atomic absorption spectrophotometer and concentration was measured by comparing the readings with the standard calibration curve. The bacterial population was counted in rhizospheric soil through serial dilution and pour plate technique [31,32].

### 4.3. Field trials

Four field trials were conducted to confirm the results from the pot study. The experiment was laid out in randomized Complete Block Design (RCBD) with three replicates having the same set of treatments as the pot trial. Before sowing, soil samples were analyzed for physiochemical attributes (Table 6). The same dose of fertilizers was applied as applied in the pot experiment. The canal water was utilized to irrigate the wheat. All agronomic practices were followed by harvesting as and when required. At maturity, growth parameters were recorded, and the crop was harvested for yield measurement. Grain samples were digested through the di-acid digestion technique and absorbance was measured on atomic absorption spectrophotometer-AAS (similar as pot trial) for Fe and Zn [30]. Rhizospheric soil samples were analyzed for the bacterial population through serial dilution and pour plate method [31].

### 4.4. Statistical analysis

Means were separated by Fisher’ protected least significance difference (LSD) at either P < 0.05 [33].

## 5. Conclusions

Enrichment of Zn and Fe to make wheat grains fortified with these deficient minerals build up a significant knowledge. The present study confirmed the promise of bio-inoculants for micronutrients fortification in shoot and grains of wheat crop. Utilization of bacterial strains *Paenibacillus polymyxa* (ZM27), *Bacillus subtilis* (ZM63), *Bacillus aryabhattai* (ZM31), and *Paenibacillus polymyxa* (S10) comprehensively contribute to making accessibility of significant nutrients particularly Zn and Fe in wheat crop. Significant improvement of nutritious minerals Zn and Fe were noted with consortia application of novel strains ZM27+ZM63+S10 compared to other inoculated/un-inoculated treatments. Novel bio-inoculants, comprising either sole or consortia led to an improvement in the plant growth parameters, besides enriching wheat grains’ nutritional status, illustrating their potential, predominantly the consortium application of ZM27+ZM63+S10. This treatment showed up to a 13% and a 15% increase in Fe and Zn content, respectively. While up to a 17% increase in grain yield of wheat was also recorded. These innovations can be suitable options for biofortification of the wheat crop with Zn and Fe through their solubilization, mobilization and translocation of nutrients to the shoot and grains by utilizing these novel strains.

## Supporting information

S1 File (PDF)
